The article "Robust method for TALEN-edited correction of pF508del in patient-specific induced pluripotent stem cells" was retracted in 2017. Reasons: no approval from an author; no approval from a third party; concerns about the data.

# Robust method for TALEN-edited correction of pF508del in patient-specific induced pluripotent stem cells

**DOI:** 10.1186/s13287-016-0275-6

**Published:** 2016-02-09

**Authors:** María Vicenta Camarasa, Víctor Miguel Gálvez

**Affiliations:** Caubet-Cimera Foundation, Hospital Joan March, Ctra Soller Km 12, 07110 Bunyola, Mallorca Spain

**Keywords:** Homologous recombination, Patient-specific stem cells, Stem cell/genetic therapy

## Abstract

Cystic fibrosis is one of the most frequent inherited rare diseases, caused by mutations in the cystic fibrosis transmembrane conductance regulator gene. Apart from symptomatic treatments, therapeutic protocols for curing the disease have not yet been established. The regeneration of genetically corrected, disease-free epithelia in cystic fibrosis patients is envisioned by designing a stem cell/genetic therapy in which patient-derived pluripotent stem cells are genetically corrected, from which target tissues are derived. In this framework, we present an efficient method for seamless correction of pF508del mutation in patient-specific induced pluripotent stem cells by gene edited homologous recombination. Gene edition has been performed by transcription activator-like effector nucleases and a homologous recombination donor vector which contains a PiggyBac transposon-based double selectable marker cassette.

This new method has been designed to partially avoid xenobiotics from the culture system, improve cell culture efficiency and genome stability by using a robust culture system method, and optimize timings. Overall, once the pluripotent cells have been amplified for the first nucleofection, the procedure can be completed in 69 days, and can be easily adapted to edit and change any gene of interest.

**Electronic supplementary material:**

The online version of this article (doi:10.1186/s13287-016-0275-6) contains supplementary material, which is available to authorized users.

## Introduction

Genetic correction by homologous recombination (HR) had proven extremely inefficient in human embryonic stem (hES) or human induced pluripotent stem (hIPS) cells before the advent of genome editing [1] and the addition of ROCK (Rho-associated, coiled-coil-containing protein kinase) inhibitor to cell dissociation steps [2]. Gene editing technologies have evolved quickly during the past 10 years. Correction of monogenic disorders in patient-specific induced pluripotent stem (iPS) cells is feasible nowadays with the aid of gene editing tools recently developed in several laboratories worldwide [3]. Efficiencies of homologous recombination increased 100-fold with the addition of engineered nucleases to edit the gene of interest [4], although the need for introducing selectable markers in the repair vector to isolate target clones persisted in order to make the correction task feasible. Even if targeted correction has been achieved in loci which are not being expressed [5], genes which are highly expressed are expectedly edited at higher frequencies [6, 7] due to the more accessible state of their chromatin.

The article "Robust method for TALEN-edited correction of pF508del in patient-specific induced pluripotent stem cells" was retracted in 2017. Reasons: no approval from an author; no approval from a third party; concerns about the data.

Gene edition with recombinant nucleases follows a multi-step procedure mainly divided into three sections: 1) creating specific double strand breaks (DSBs) by engineered nucleases, near to the desired locus on the genome; 2) triggering the homology-directed repair (HDR) process and editing the gene by means of adding a donor vector with homology arms and selectable markers as a repair template for homologous recombination; and 3) seamlessly removing selectable markers from isolated clonal or semiclonal populations. Repair template contains homology arms matching 5’ and 3’ regions surrounding the DSB point. Selectable markers are needed to identify successfully corrected genomes. The rationale behind this repair has been highly argued and readers are referred to the literature for a detailed explanation [8].

At present, there are three major kind of engineered nucleases: zinc finger nucleases (ZFNs), transcription activator-like effector nucleases (TALENs), and clustered regularly interspaced short palindromic repeats/associated (CRISPr/Cas) nucleases [9]. All these nucleases contain an encoded recognition mechanism and a nuclease (Fok I or Cas9). TALENS have been reported to be more efficient than ZFNs [10], and generation of off-target mutations by TALENs have also been found to be fewer [11]. The construction of guide RNAs in CRISPr/Cas nucleases has been developed to a simple and efficient procedure [12] but lacks the heterodimerization safety mechanism shared by ZFNs and TALENS [13], which implies the recognition of two different targets in order to promote a DSB event.

Elimination of the selectable markers after genetic repair with most common Cre/loxP, Flp/FRT, and ϕC31 integrase/attP-attB recombination systems leave small ectopic sequences in the genome, which even if located in intronic regions could have the potential to interfere with transcriptional regulatory elements [14], splicing machinery, or cause unexpected translocations and genome reorganizations [15].

The addition of transposons/transposase as an alternative to the list of recombinase mechanisms [16] has constituted a second milestone after the engineered nucleases for completing genome edition in a seamless manner. Transposons are well known to work in mammalian cells and transposases produce safer elimination of the selectable cassettes without altering genomic DNA sequence. PiggyBac transposon has been proven to efficiently transpose in mammalian cells including hES cells [17, 18]. The strategy of introducing a double selectable marker gene (*puroΔtk*) in a transposon in the repair vector was developed previously and applied to the correction of A1AT deficiency in patient-specific iPS cells [19]. After homologous recombination, transposase is transgenically expressed and carries out the excision of the selectable cassette from the repaired clones by recombination between head and tail (PB) sequences. The excision overrides a TTAA motif—AA from the transposon head and TT from the transposon tail—which leaves an intact genome if it has been integrated at a TTAA site as is the case in our work. Interestingly, the hyperactive transposase has double efficiency for excision rather than for integration, which is a convenient trait and another reason for having chosen this system for cystic fibrosis transmembrane conductance regulator (CFTR) gene repair [20].

The article "Robust method for TALEN-edited correction of pF508del in patient-specific induced pluripotent stem cells" was retracted in 2017. Reasons: no approval from an author; no approval from a third party; concerns about the data.

Cystic fibrosis (CF) is one of the most frequent rare diseases, caused by mutations in the CFTR gene. Apart from symptomatic treatments, there is no alternative to cure the disease at present [21]. Recently, the correction of the pF508del mutation in patient-specific iPS cells has been published [22, 23], and confirmation of the production of the wild-type protein by the corrected cells has been performed after directed differentiation to intestinal epithelial cells. In our case, the differentiation of pluripotent repaired cells to airway and intestinal epithelial cells has been performed to confirm functional restoration of the CFTR channel and data will be published elsewhere as it is beyond the scope of this method of genetic correction by TALEN-edited homologous recombination.

In the present work, we designed and constructed a PiggyBac-based HR vector, and nucleofected it in combination with TALENs specifically designed to cut in the region near the CTT (pF508del) deletion of the human CFTR gene. Positive selection of the recombinant clones was performed by resistance to puromycin, and polymerase chain reactions (PCRs) designed to detect the integration of vector homology arms were conducted on genomic DNA from all of them. Hyperactive transposase was transfected in a list of more than ten positively targeted clones, and upon transposon removal a negative selection for *Tk* expression was conducted by treatment with fialuridine (1-(2-deoxy-2-fluoro-1-D-arabinofuranosyl)-5-iodouracil; FIAU), an analog of ganciclovir. Surviving clones were expanded and checked by PCR for elimination of the selectable cassette, and CFTR alleles were cloned and sequenced on several of them to identify successfully repaired patient-specific CFTR^pMC3.1/pF508Δ^. One hIPS cell line from each of two patients was corrected. CF is a monogenic recessive disease, therefore heterocygotic correction is sufficient to restore CFTR function in repaired cells.

The article "Robust method for TALEN-edited correction of pF508del in patient-specific induced pluripotent stem cells" was retracted in 2017. Reasons: no approval from an author; no approval from a third party; concerns about the data.

## Methods

There are seven major stages in the correction of disease-associated genetic mutations by TALEN-edited seamless HR in patient-specific pluripotent cells: 1) the generation of patient-specific iPS cells including confirmation of the mutation and its homo- or heterocygosis; 2) the design and construction of the nuclease and the donor vectors for HR; 3) the repair experiment itself with selected nucleases according to their cutting efficiency and the preparation of replicated cultures of positively selected populations; 4) the design and carrying out of the PCR screening to assess positive candidates; 5) the elimination by transposition of the selectable double marker in chosen candidate populations and negative selection procedure; 6) the cell cloning and screening of selected populations for the effective elimination of the selection cassette; and 7) the confirmation of the bona fide correction and the absence of other unwanted genetic modifications in chosen repaired clones.

Patient-specific hIPS cell line establishment and characterization has been performed according to the work already described elsewhere [24, 25]. In this method, we describe stages 2 to 7 of the genetic correction of pF508Δ mutation in two of the reprogrammed hIPS lines. Methodology for completion of each step is detailed in the following sections.

### Design and construction of the donor/targeting vector

ZFN expression vectors were originally designed using ZiFiT targeter software provided by the Zinc Finger Consortium (http://zifit.partners.org). CompoZr® Knockout ZFN, engineered ZFNs for pF508Δ targeting from Sigma™, were supplied under a collaboration agreement. TALEN vectors designed to cut in the same spot as ZFNs were designed and purchased from Transposagen®.

pMC3.1 donor vector was designed as a unique sequence and synthesized. Two homology arms of 916 base pairs upstream and downstream of the DSB spot were included, respectively, with five silent point mutations at the 3’ side of the 5’ homology arm designed in order to: a) create a restriction site (for BglII as it has unique cutting site in the whole recombination region) which will be useful in the identification of the recombined alleles during screening; b) avoid recognition of the recombined allele for the nucleases (re-targeting); and c) design specific primers for the recombined allele versus the endogenous ones. Besides the homology arms, the synthetic (control) vector designated as Seq_1 contained homology arms surrounded at 5’ and 3’ ends by specific genomic regions chosen as primers for PCR detection of recombination events, respectively. EcoRI and MluI sites were designed at both ends of each string, respectively, so they could be easily eliminated from the control vector during construction of the targeting vector.

The article "Robust method for TALEN-edited correction of pF508del in patient-specific induced pluripotent stem cells" was retracted in 2017. Reasons: no approval from an author; no approval from a third party; concerns about the data.

Construction of the donor vector for HR experiments was thus performed in three steps of modification of this synthetic control vector: first, EcoRI digestion of Seq_1 eliminated the contiguous genomic region in the 5’ arm (generating Seq_2); then MluI digestion eliminated the contiguous genomic region in the 3’ arm (Seq_3); in the third step, digestion of the NheI/NotI fragment from the pMCS-AAT-PB:PGKpuroΔtk vector was cloned into NheI/NotI sites in Seq_3, introducing the PuroΔtk/PiggyBac (PB) transposon cassette in between the homology arms to generate the donor targeting vector pMC3.1 (Seq_4). PMCS-AAT-PB: PGKpuroΔtk is the targeting vector used for A1AT correction [19] and was obtained from the Sanger Institute (http://www.sanger.ac.uk/form/-C3ZIws9wQ4CSysnb1AY4kA) under an MTA agreement.

The pMC3.1 targeting vector, besides having a strong double selection cassette, allows for screening strategies for each step of the HR procedure: PCR amplification for positive recombinant clones, restriction fragment analysis of the recombinant allele to check the stability of its open reading frame (ORF), and detection of the reverted allele after excision of the transposon/selection cassette, when we can use the point mutations located at the nuclease recognition sites to amplify specifically recombined and non-recombined (either mutated or corrected) alleles. This screening system shares a common forward primer and uses two different reverse primers which will recognize native from recombined alleles.

### Nuclease efficiency assessment

CelI assay [26, 27] for detection of mutations was used to estimate the cutting efficiency of ZFN and TALEN nucleases used in this work. The rationale behind this method of detection of nuclease activity is the generation of mismatches in the genomic DNA as a consequence of natural cellular repair of a DSB in the absence of homology templates. This mechanism of repair is known as non-homologous end-joining (NHEJ) and the celery enzyme CelI was found to cut dsDNA at mismatches but not at paired bases. After PCR amplification of the fragment, digestion confirms the presence of repaired DNA at that site, which implies previous DSB generation and repair by NHEJ. Surveyor assay kit® from Transgenomic® was used following the manufacturer’s instructions. Briefly, K562 and CFhIPS3.18 were nucleofected with 2 μg of each nuclease plasmid and cells were cultured for 48 hours. Genomic DNA was extracted, digested, and run on agarose gels. Results were obtained by densitometric quantification of digested versus undigested bands, using the formula 100 × cleaved/cleaved + parental.

The article "Robust method for TALEN-edited correction of pF508del in patient-specific induced pluripotent stem cells" was retracted in 2017. Reasons: no approval from an author; no approval from a third party; concerns about the data.

### Cell culture and characterization

hIPS cell lines were generated and described elsewhere [26]. Briefly, CFhIPS3.18 and CFhIPS4.4 were cultured on human foreskin fibroblasts, HFF-1 feeder layers with HESNEW_S media containing KO DMEM supplemented with 20 % knockout serum replacement, 1 mM GlutaMax, 0.1 mM 2-mercaptoethanol (2-ME), 1× non-essential amino acid and 8 ng/ml of fibroblast growth factor 2 (FGF2). All cultures were performed without the addition of antibiotics. Subculture was performed mechanically for up to eight passages during line derivation, and then recombinant trypsin was used in combination with ROCK inhibitor to produce near-single cell suspensions (i.e., small clumps of 5–20 cells, approximately). Established pluripotent lines were characterized for stemness, pluripotency and genetic stability during continuous expansion in culture following basic protocols with slight modifications as described previously [28]. Stem cell markers were detected by immunofluorescence in pluripotent colonies, and pluripotency markers were detected after spontaneous differentiation of embryoid bodies (EBs) for 10–12 days in suspension cultures on SBF-containing medium, previously to continuous 25–30 days in adherent cultures in the same medium. Instead of in vivo differentiation by teratoma formation, a novel method of three-dimensional culture of EBs was assayed on Aggrewell® plates. After a month of continuous culture, mature EBs were paraffin-embedded and sectioned for immunohistochemistry staining following a standard procedure. One line from each patient was chosen to perform homologous recombination experiments.

### Gene targeting in CFhIPS lines

CFhIPS3.18 and CFhIPS4.4 were nucleofected with ZFN and pMC3.1 plasmids at a ratio of 1 μg of each ZFN and 2 μg of the targeting vector per million cells. For TALEN experiments, TALENs and donor vector were mixed and nucleofected at a ratio of 2 μg of each circular vector per million cells using an Amaxa nucleofector device II and following manufacturer instructions. After nucleofection, hIPS cells were seeded onto HFF-1/W3R feeders [29], kindly provided by Dr Chen at the Johns Hopkins University School of Medicine in Baltimore, MD, USA. These cells are resistant to neomycin, hygromicin and puromycin, allowing selection for the expression of the PuroΔ*tk* cassette. Briefly, subconfluent cells were trypsinized and resuspended in HESNEW medium containing ROCK inhibitor before centrifugation at 200 g and resuspension in nucleofector solution 2 (and lately equivalent P3 due to commercial availability). B16 program was used for best results combining nucleofection efficiency and cell viability. Nucleofected cells were plated onto resistant feeders described before in the presence of ROCK inhibitor for 1 day in HESNEW_S, and thereafter the media was substituted by the puromycin-containing HESNEW_R at 1 μg/ml. Emerging resistant clones were allowed to grow and subcultured individually up to 16 days after plating, feeding them every second day. Grown colonies were manually picked and transferred to 48 tissue culture microplates, which were grown for an additional 5 to 8 days. Clones were then replicated by trypsinization, and grown until at least 50 % confluence. One replica plate was frozen and the other was used for genomic DNA extraction which was performed manually by a basic protocol. Briefly, cells were lysed in high salt content buffer and genomic DNA was precipitated with isopropanol and washed in ethanol before resuspension in Tris-EDTA buffer.

The article "Robust method for TALEN-edited correction of pF508del in patient-specific induced pluripotent stem cells" was retracted in 2017. Reasons: no approval from an author; no approval from a third party; concerns about the data.

### PCR screening and Sanger sequencing

Genomic DNA from 48-well replica plates of colonies resistant to puromycin was extracted by proteinase K digestion of the cells on the plate by lysis buffer and precipitation of the DNA with isopropanol after transferring lysates to eppendorf tubes. DNA pellets were washed in 70 % ethanol and resuspended in Tris-EDTA buffer. PCRs were performed at annealing temperatures according to temperature gradient optimization for each pair of primers, and extension times according to product length (see Table 1). Table 2 shows detail of the chemistry of the PCRs according to product length. Genotyping PCRs were performed for both recombination arms. Primers for amplification of the homology arms were located in the genomic region (5’ on the 5’ arm and 3’ on the 3’ arm, respectively. PCR screening for both arms plus BglII digestion pattern were used to assign positive clones for homologous recombination (Fig. 1 depicts the scheme of the repair strategy). Primers used for each step of the screening are indicated as arrowheads in Fig. 1 and their sequences are listed in Table 3.

**Table 1:** PCR conditions for genotyping after nucleofections in repair experiment

‘SHORT PCR’ 351/406 bp DSB target/reverted allele	‘MED PCR’ 1234/1346 bp Homology arms	‘LONG PCR’ 2360/2509 bp Full endogenous/reverted allele
95 5’	95 5’	95 5’
95 30”	95 30”	95 30”
64 15”	64 45”	64 45”
72 30”	72 2’	72 3’
40 cycles	40 cycles	40 cycles
72 7’	72 7’	72 15’

*bp* Base pair, *DSB* Double strand break, *PCR* Polymerase chain reaction. Left numbers on each cell of the table correspond to Temperatures, and right numbers correspond to times for each step of the PCR amplification

The article "Robust method for TALEN-edited correction of pF508del in patient-specific induced pluripotent stem cells" was retracted in 2017. Reasons: no approval from an author; no approval from a third party; concerns about the data.

**Table 2:** PCR reaction chemistry

		SHORT PCR		MED/LONG PCR	
	Working dil	Final conc./rxn	μl/25 μl	Final conc./rxn	μl/25 μl
DNA seq-1 696.9 ng/μl	10^−3^/10^−6^	≈300 ng	2.0 μl	≈300 ng	2.0 μl
Primer up	10 μM	0.4 μM	1.0 μl	0.4 μM	1.0 μl
Primer dwn	10 μM	0.4 μM	1.0 μl	0.4 μM	1.0 μl
dNTPs	2.5 mM	100 μM	1.0 μl	200 μM	2.0 μl
Buffer 10×	10×	1×	2.5 μl	1×	2.5 μl
MgCl_2_	50 mM	3 mM	1.50 μl	2 mM	1.0 μl
Taq	5 U/μl	2.5 U	0.5 μl	0.5/1/2.5 U	0.5 μl
H_2_O			15.5		15

*PCR* Polymerase chain reaction; *dil* dilution; *conc* concentration; *rxn* reaction; *dNTPs* deoxynucleotides triphosphates mixture; *dwn* down (3' end)

**Fig. 1:** **a** Schematic drawing of the genomic edition and HR steps to correct pF508del mutation. After specific cut by ZFNs or TALENs, repair vector is used as a template for homologous recombination and the process generates the P allele, which shows homology arms and position of the primers (P3–4 and P5–6) used for their amplification and detection, with one primer 5’ or 3’ in the genomic region and the other 3’ or 5’ in the terminal repeats of the transposon cassette, respectively. Transposase is then expressed in target cells to eliminate the double selectable marker, which has sequentially selected cells resistant to puromycin which have integrated the donor vector and, from these, cells resistant to Fialuridine which have eliminated the transposon containing the modified Thymidine kinase gene in sequential steps. Primers P1–2 allow for confirmation of the repaired sequence. **b** Genomic sequence detail of the targeting region, showing the position of the pF508del mutation, ZFN and TALEN target sequences and spacers, silent mutations introduced to avoid retargeting and to create a restriction site to distinguish targeted allele, and TTAA position for the introduction of the PiggyBac double selectable marker. *TALEN* Transcription activator-like effector nuclease, *ZFN* Transcription activator-like effector nuclease

**Table 3:** Sequences of primers used in each step of screening for positive and negative selection steps during edited genome repair

CR4 Up	TAG GTT GTA GCA GTG GTA GTG
CR4 Down	CTC TAT GTA ACT CTT GTC TCT TCC
ZFN F	TGG AGC CTT CAG AGG GTA AA
ZFN R	TTT CAT GTG TTT GCA AGC TTC T
Integra5.1up	TCC TCT GCT ACC TCC TTT CCT TCT
Integra5.2up	TCT TCC TCT GCT ACC TCC TTT CCT
Integra5.3up	TGC TTT TTC TTC CTC TGC TAC CTC C
Integra5.4up	TTC CTC TGC TAC CTC CTT TCC TTC T
Integra5.5up	TCC TCT GCT ACC TCC TTT CCT TC
Integra5.1dn	GGA GCT CCA AGC GGC GAC TG
Integra5.2dn	GCC TCA CGG GAG CTC CAA GC
Integra5.3dn	TGA CAA GCA CGC CTC ACG GG
Integra5.4dn	CTC ACG GGA GCT CCA AGC GG
Integra5.5dn	ACC GCA TTG ACA AGC ACG CC
Integra3.1up	ACA GAC CGA TAA AAC ACA TGC GTC A
Integra3.2up	CAG ACC GATA AAA CAC ATG CGT CA
Integra3.3up	AGA CCG ATA AAA CAC ATG CGT CA
Integra3.4up	CAG ACC GAT AAA ACA CAT GCG TCA A
Integra3.5up	AGA CCG ATA AAA CAC ATG CGT CAA
Integra3.1dn	AGG CAC CTT CCG CAA CTT TTC CA
Integra3.2dn	GGC ACC TTC CGC AAC TTT TCC A
Integra3.3dn	AGG CAC CTT CCG CAA CTT TTC C
Integra3.4dn	GGC ACC TTC CGC AAC TTT TCC AC
Integra3.5dn	GGC ACC TTC CGC AAC TTT TCC
Reint F	CTG CTG CAA CTT ACC TCC GGG ATG
Reint R	CCA ATC CTC CCC CTT GCT GTC CTG
Recomb F	TCT GTC ATC AAA GCC TGT CAG C
Recomb R	GCTCGTTGACCTCCACTCAG
ENDO F	GCGTCATCAAAGCATGCCAAC
PB-out-F	GATCTGTCATCAAAGCCTGTCAG
PB-out-R	CAGATCAATGCTCATTCCATTAGGC

After correction, two rounds of PCR were performed to confirm the absence of reintegration of the PiggyBac double selectable marker cassette. First, Recomb F/ZFN R primers were used to check for correct size of the targeted fragment after cassette excision in the edited allele (i.e., in the original place), and then Reint primers were used to confirm that no random reintegration of the transposon occurred in the genome.

The article "Robust method for TALEN-edited correction of pF508del in patient-specific induced pluripotent stem cells" was retracted in 2017. Reasons: no approval from an author; no approval from a third party; concerns about the data.

### Transposon excision in CFhIPS/ ^pMC3.1^ sub-lines

Confirmed positive clones for HR were thawed and expanded, and subjected to cassette excision by nucleofection of 5 ug of the pCMV-HAhyPBase vector that encodes the transposase per million cells. FIAU selection was applied from day 1 onwards after nucleofection, and resistant clones were mechanically split and subcultured for at least three passages until genomic DNA was extracted for analysis. After FIAU selection for *Tk* negative events resulting from the elimination of the selectable cassette, resistant colonies were isolated and duplicated in P48 well plates. One replica was expanded in culture while the other was used for PCR screening and DNA sequencing. CFTR alleles were cloned and sequenced in both senses with 5’ and 3’ primers separately, and reactions were purified with a column and sent to Secugen®. Results were visualized in Chromas software and browsed in GenBank for identity check.

### PROGNOS and array comparative genome hybridization

Stage 7 of DNA repair, which is confirmation that no other mutations have been generated during the repair procedure, was completed by PROGNOS software and Sanger sequencing of the predicted off-target sites. Predicted Report Of Genome-wide Nuclease Off-target Sites (PROGNOS) online software from Gang Bao laboratory was used to evaluate potential rearrangements in off-target sequences throughout the genome after pF508Δ correction by HR [30]. Target sequences for both TALENs, variable length of the spacer from 10 to 30 bases, and precise repeat variable domains (RVDs) of the TALENs were used to interrogate PROGNOS for possible off-target sequences. Genomic DNA extracted from corrected clones was used as a template for PCR amplification of predicted off-target loci with primers designed by the same software. Sanger sequencing of the products was performed to check for the absence of mutations which would have been expected as a result of NHEJ events after putative unspecific cut by TALENs.

The article "Robust method for TALEN-edited correction of pF508del in patient-specific induced pluripotent stem cells" was retracted in 2017. Reasons: no approval from an author; no approval from a third party; concerns about the data.

The same genomic DNA from corrected lines was submitted to comparative genome hybridization array (aCGH) analysis (outsourced).

## Results and discussion

### Generation and characterization of patient-specific hIPS cell lines

A panel of ten hIPS lines was established from keratinocytes and fibroblasts of two CF patients and one healthy donor (in preparation). Stable pluripotent lines were continuously cultured and expanded to prepare frozen stocks at low passages (6–15). Additional file 1 (Figure S1) and Additional file 2 (Figure S2) show representative results of the immunofluorescence for stemness and pluripotency markers in several of the lines analyzed from each patient. Genetic stability was assessed by karyotype every ten passages, and was found to be normal in all ten lines tested up to passage 42. Additional file 3 (Figure S3) shows the karyotype of hIPS3.18 and hIPS4.4 at the same passage that was used for the HR experiment. Tissue formation from all three germ layers was assessed by hematoxylin and eosin staining in sections of paraffin-embedded EBs cultured for more than a month, following a novel protocol whose results are equivalent to teratoma formation in mouse models (Additional file 4: Figure S4).

Basic human pluripotent culture is best routinely maintained in parental HFF-1 fibroblasts which are irradiated at 40 Gy and frozen as batches of around 180 million cells each in vials of 2–3 million cells each. Growth and amplification of resistant populations is then best achieved using resistant human fibroblasts, which are robust feeders during the relatively long period of culture for clonal growth of rare events, as positive recombinants. With this system, feeder supplementation is avoided at any time and pluripotent culture is robustly supported.

### TALEN cutting efficiency

Efficiency of CompoZr® CFTR_ZFN was calculated to be 12.4 % by Sigma in the K562 human promyelocytic leukemia cell line. Surveyor assay for TALENs resulted in a cutting efficiency of 2.76 % in one of our CFhIPS pluripotent cell line (see Additional file 5: Figure S5 for an image of electrophoresis results of Surveyor assay in oneCFhIPS line). This discrepancy and lower cutting efficiency for TALENs could be attributable to the differences in efficiency of nucleofection between the two cell types which are widely known. Nucleofection efficiency in human pluripotent stem cells is known to be significantly lower than in mouse pluripotent stem cell lines and in other cell types in general.

The article "Robust method for TALEN-edited correction of pF508del in patient-specific induced pluripotent stem cells" was retracted in 2017. Reasons: no approval from an author; no approval from a third party; concerns about the data.

### Correction of pF508Δ in patient-specific hIPS cell lines

Fibroblasts from two CF patients were reprogrammed to pluripotency by viral-driven expression of the four Yamanaka factors. Homocygous pF508 deletion was confirmed by digestion PCR as previously published [31], and Sanger sequencing, in both original fibroblasts and resulting pluripotent lines. From a panel of derived lines, CFhIPS3.18 and CFhIPS4.4 from each patient, respectively, were nucleofected with a pair of TALEN and a donor vector designed to introduce a CTT to restore pF508Δ mutation. Figure 1a shows the diagram of the strategy for correction of the mutation. The original mutated allele in exon 11 of CFTR would be cut by ZFN or TALEN recombinant nucleases in the presence of the targeting vector, which would have generated the P allele by homologous recombination. A transposon vector containing the double selectable marker PuroΔtk was chosen for the possibility of seamless excision of the cassette after correction. After assignation of positive targeted clones by PCR using primers depicted as arrows in the diagram, nucleofection of the hyperactive transposase would restore genomic sequence to the corrected/edited one. Silent mutations created a BglII site in the left homology arm to aid in the identification of the edited allele. Additional silent mutations were introduced in the targeting vector in the recognition sites for ZFNs and TALENs to avoid retargeting as well, as indicated in Fig. 1b. The indicated TTAA marks the position of integration of the transposon. A ZFN and a TALEN pair of recombinant nucleases were designed to target the same locus, and homologous recombination experiments were performed with both using the same targeting vector with a transposon-based double selectable marker. Under continuous puromycin selection, 1318 resistant clones were screened by PCRs for 5’ and 3’ arms respectively after nucleofection of ZFNs + pMC3.1 vectors into the CFhIPS3.18 line, with no positive result for a recombination event. ZFN vectors targeting the same region had been used before with similar results of no demonstrated correction [32].

Efficiencies of recombination for the pMC3.1 repair vector in combination with TALEN plasmids are shown in Table 4 for two CFhIPS lines, each one corresponding to each donor patient studied. Figure 2a and b shows examples of PCR results for detection of 5’ and 3’ homology arms, respectively. Digestion with BglII was performed on an aliquot of 5’-arm PCR to confirm the recombinant P allele origin of the amplified DNA (Fig. 2c), and resulted in the first indication that correction occurred only in one allele by the uncut band. Selected positive clones were nucleofected with HAHypBase vector to eliminate the PiggyBac transposon with the double selectable marker cassette. Resistant populations to FIAU were isolated and cloned, and PCR screening was performed to confirm positive events of elimination of the selectable marker (Fig. 2d), completing the correction of the pF508Δ mutation in respective hIPS lines from the two patients assayed.

The article "Robust method for TALEN-edited correction of pF508del in patient-specific induced pluripotent stem cells" was retracted in 2017. Reasons: no approval from an author; no approval from a third party; concerns about the data.

**Table 4:** Efficiencies of targeted correction of pF508del in CFhIPS lines

Line	Cell number	Puro	PCR targets	Ratio PCR targets	Efficiency
CFhIPS3.18	122 × 10^6^	648	60	9.26 %	4.9 × 10^−5^
CFhIPS4.4	58 × 10^6^	98	10	10.20 %	1.7 × 10^−5^

*PCR* Polymerase chain reaction

**Fig. 2:** PCR screening steps for detection of pF508 correction. **a** Ethidium bromide stain of the gel showing positive amplification of the left homology arm of the targeted P allele. **b** In a similar fashion, gel image showing positive clones for amplification of the right arm. In both **a** and **b**, positive PCR reactions correspond to PCRs performed with same test primers on the control vector as a template, which contains adjacent genomic sequences to the 5’ end of the 5’ arm and the 3’ end of the 3’ arm. **c** BglII cut of the 5’ arm, confirming the presence of P recombined allele on positive clones. **d** PCR result of the targeted region after elimination of the selection cassette by transposase expression. Band size confirms elimination of the transposon-based double selectable marker from the homologous integration site

After confirming correction and elimination of the selection cassette from the designated clones, DNA sequencing was performed on the full recombination region on cloned alleles to confirm positive correction/addition of the CTT to the original mutated sequence in heterozygosis, and absence of additional mutations in the region. Figure 3 shows lack of CTT on one of the cell lines corrected (Fig. 3a) and CTT addition on Sanger sequencing electropherogram of genomic DNA after edited repair (Fig. 3b). In Fig. 4, fragments of the edited/corrected alleles in both lines are annotated. CTT presence along with Bgl-II introduction and silent mutations are indicated. Full sequences in Additional files 3 and 4 contain the sequencing pattern and alignments of the full homology fragments after repair in both lines assayed. Correction of the mutation resulted in heterocygosis in all sub-lines analyzed.

The article "Robust method for TALEN-edited correction of pF508del in patient-specific induced pluripotent stem cells" was retracted in 2017. Reasons: no approval from an author; no approval from a third party; concerns about the data.

**Fig. 3:** Sanger sequencing on negatively selected clones after correction of pF508del mutation. **a** Representative genomic electropherogram of CFhIPS3.18, showing the point of the deletion. **b** Genomic sequence electropherogram after homologous recombination and marker transposition, showing CTT addition which means correction of the deletion causing CF

**Fig. 4:** Annotated DNA sequences of the edited alleles in both corrected CFhIPS lines. Annotated sequences of edited alleles in **a** CFhIPS3.18 and **b** CFhIPS4.4. The BglII site created de novo and the rest of silent mutations introduced to avoid nuclease retargeting are indicated in the panels

### Off-target analysis and aCGH

After confirming correction of the mutation by Sanger sequencing, PROGNOS software was used to predict off-target sequences of the nucleases throughout the genome. PROGNOS results are summarized in Table 5. Mismatches required for off-target cut by the TALEN pair used in this work are detailed in column 3, for the 5’ TALEN or for both. PCR primers given by PROGNOS for all 15 off-target sites are listed in Table 6. Genomic DNAs from repaired and sequenced clones included in Fig. 4 were used for sequencing of the PCR amplicons suggested by PROGNOS, with the result of wild-type sequences in each case (in preparation, data not shown). Comparative genome hybridization between parental and edited lines resulted in no relevant genomic alterations due to the TALEN-edited targeted correction of pF508Δ (in preparation).

**Table 5:** PROGNOS results for prediction of pF508del_TALENs off-targets

Ranking	Hom.	Mismatches	Chromosome_Name	Genomic_Region	Closest_Gene
1	98	0_0	chr7	Exon	CFTR
2	37	6_1	chr4	Intergenic	TECRL
3	26	6_2	chr9	Intron	PALM2-AKAP2
4	17	6_3	chr19	Intergenic	ZNF714
5	26	6_2	chr17	Intergenic	NLRP1
6	17	6_3	chr13	Intergenic	LINC00550
7	25	4_3	chr9	Intron	MPDZ
8	17	6_3	chr2	Intergenic	KCNE4
9	18	4_4	chr9	Intergenic	MAMDC2
10	17	6_3	chr8	Intergenic	FGF20
11	26	6_2	chr6	Intergenic	KIAA1009
12	17	6_3	chr6	Intron	CDKAL1
13	18	4_4	chr3	Intergenic	TMEM207
14	17	6_3	chr13	Intron	ATP11A
15	20	5_3	chr8	Intergenic	WRN
16	13	5_4	chr4	Intergenic	PDHA2

**Table 6:** Primers inferred by PROGNOS algorithm for TALEN pair off-target check

R.	S.	Forward_Primer	Reverse_Primer
1	98	GGCAAGTGAATCCTGAGCGTG	CATTCACAGTAGCTTACCCATAGAGGAAAC
2	37	CTGTCAAAGTGGGCTCCTATTTGC	CAGACATGTCAAAAAGATGCTGCCCAGA
3	26	GGGTAGCAGCGAAACAGAAAAGG	GGCAACACAGTGAGACTCCATC
4	17	CTGCTCCATTGGCCTATATCTCTG	CAAACTGACTCCAGTGAGATGGTG
5	26	CTTTTGGTGGCGAAATAGGGGTG	CTTATGCATGCGCACCCATGTAC
6	17	GAAGATAGGGAACACCTACTGACAAGTCAT	CCTTCCACTGTTTCTTTCCTATATTCTTGTCC
7	25	GGAAAGACAGTAGTCATCTCCCC	CCAGGACATGTCTGAGGAGTCT
8	17	GCCTAAATCCAACATTATACTAGATGTCCC	GATCTGCATGCTGCTTCTGCC
9	18	GGAGCATGGTTGCTGGATCATAC	CACAGGCTGCTCTTGCAAAAACAC
10	17	CCTGGCTGCCTCTTTGACTG	GCCACTTTCCTGAGAAGAACTGC
11	26	GGATGTGGCTCCTGGGTTTTTAG	GTAACCACATGCCTAGAGGGTAGT
12	17	CATGAGTCTCCAGACTGTACCTTG	CACTCCTTTCAGGTGTGTGTTGC
13	18	GGCACCAAGAACATACAACAGGG	GCTGTGGAGTTGTGTGAGCTCT
14	17	AGCATAGCACTGGAAGCTCTAGCC	CCTCTGGACACAAATCCAGTCAGT
15	20	GGAGCTGGTGTCACTGCAGA	GACTGCCCAAAATCAAGCGTGGT
16	13	GGAGCTACAGTTAGGGTGCAATTC	GTTGCCAGAAGGCAGAATTAGGAG

The article "Robust method for TALEN-edited correction of pF508del in patient-specific induced pluripotent stem cells" was retracted in 2017. Reasons: no approval from an author; no approval from a third party; concerns about the data.

## Conclusions

It is well established that a feeder-based culture is better than feeder-free culture methods to maintain karyotypic stability on human pluripotent stem cells [33]. The presently described culture system is designed to avoid xenobiotics as much as possible whilst maintaining basic culture conditions for pluripotent cells, i.e., a feeder-based cell culture system, which is known to maintain genomic stability for a larger number of passages compared to feeder-free systems [34]. The use of human parental and human resistant feeder sub-lines allowed for robust cultures which were easily scalable and frozen/thawed, adding versatility to the technology and, overall, posing less stress to cells in terms of genomic stability. The HFF-1 human foreskin fibroblast line from ATCC and the HFF-1/W3R Wnt expressing sub-line have proven robust tools in the design of the culture protocol for the different steps of the procedure. HFF-1/W3R is resistant to neomycin, hygromycin and puromycin. Moreover, the use of continuous lines as feeders as opposed to traditional primary mouse embryonic fibroblasts adds reproducibility and reduces workload. In conclusion, the method chosen in this protocol with the use of parental human foreskin fibroblasts and resistant sub-lines for homologous recombination experiments has proven robust and has allowed the achievement of genetic correction in about 2 months, a shorter period compared to other protocols [19].

In previous HR strategies, the removal of the selection cassettes left residual sequences in the edited locus, which although placed more often in the intron part of the edited gene implied locus restrictions for HR strategies. The new strategy using transposon/transposase as the recombination method avoids the introduction of foreign sequences in the recombinant allele. Furthermore, the pMC3.1 vector, apart from having a strong + (puro)/–(Δ*tk*) PB selection cassette, offers three different screening strategies. The first one is a PCR amplification of each recombined homology arm that only will be positive once the recombination is achieved. In these PCRs, clones that are positive for 5´ and 3´ hybrid sequences were detected. The second screening implies the digestion of the 5’ arm with Bgl-II and their sequencing, in order to check the stability of the CFTR ORF. The third screening step was performed after cassette excision, where silent mutations introduced to avoid nuclease retargeting after correction were used to design a three-primer PCR system that will amplify distinctively the non-recombined alleles (wild-type (wt) used as a PCR-positive control and pF508Δ) from the recombined allele. This screening system shared a common forward primer and was based in two different reverse primers that recognized and amplified the native *CFTR/CFTRpF508Δ* (wt/mutated) allele or the recombinant *CFTR/pMC3.1* (wt/edited) allele.

The article "Robust method for TALEN-edited correction of pF508del in patient-specific induced pluripotent stem cells" was retracted in 2017. Reasons: no approval from an author; no approval from a third party; concerns about the data.

The use of TALEN-mediated HR in combination with a transposon-based double selectable marker achieved correction of pF508Δ mutation in hIPS lines from two patients at efficiencies ranging 1.7-4.9 x 10^−5^, resulting in a feasible protocol in terms of both workload and timing. Raw data corresponding to the homologous recombination experiments was communicated at a symposium organized by the Spanish Society of Gene and Cell Therapy, and is available online at http://www.setgyc.es/home/ZFN_3_M_Camarasa.pdf.

Development of generations of hIPS cells towards clinical production have been reviewed [35]. The present method improves previous endogenous genetic corrections performed in patient-derived stem cells in the following aspects: a) pluripotent cell culture is performed with minimal xenobiotic components and without the addition to antimicrobe antibiotics; b) correction is performed in a feeder-based cell culture system, which is known to offer more robustness and stability; c) repair vector has been designed as a transposon with a double selectable marker, which facilitates the processes of selection and seamless elimination of the selection cassette; and d) PCR screening has been designed to discern the endogenous from the modified allele, both either wild-type or mutated. Overall, the method described allows correction of patient-specific induced pluripotent cells in less than 3 months, and corrected cells have been directly cultured in a format which allows rapid scaling up for downstream applications.

## Additional files

Additional file 1:
**Immunofluorescence detection of stem cell markers in CFhIPS cell lines.** Immunostaining for stem cell markers in ten of the 49 lines originally generated. Markers are indicated in the panel and are distributed in columns. Lines 1 to 10 from top to bottom are designated in the panel as well. From ten lines analyzed, one presented a chromosomal anomaly and its name is depicted in red. (TIF 856 kb) Additional file 2:
**Immunofluorescence detection of pluripotency markers in ten CFhIPS cell lines.** Ectoderm (nestin, Tuj-1), mesoderm (eomes, A-actinin) and endoderm (Sox 17, GATA4) markers are shown in the ten lines fully characterized for this project. (TIF 757 kb) Additional file 3:
**Karyotypes of CFhIPS cell lines corrected for pF508del.** G-bands of CFhIPS3.18 and CFhIPS4.4, respectively, as indicated in the panels. Both lines are karyotypically normal. (TIF 1037 kb) Additional file 4:
**Histological stain for in vivo pluripotency assessment. Mallory’s tetrachromic staining of paraffin embedded embryoid bodies (EBs) derived from CFhIPS3.18.** (**A**) Different types of tissues could be found in the EBs including (**B**) columnar epithelium (endoderm), (**C**) cartilage (mesoderm) and (**D**) cuboidal and squamous stratified epithelium (Ectoderm). Scale bars: **A**, 100 μm; **B**–**D**, 50 μm. (TIF 521 kb) Additional file 5:
**Surveyor mutation detection assay to estimate TALEN cutting efficiency.** The full homology arm containing the cutting sequence was amplified and digested with CelI and T7 endonucleases as indicated in the panel. Expected size of digested bands after cut is indicated to the right and restriction fragment size marker bands are indicated to the left. Densitometric analysis of the image resulted in an indel frequency of 2.76 %. (TIF 1104 kb)

The article "Robust method for TALEN-edited correction of pF508del in patient-specific induced pluripotent stem cells" was retracted in 2017. Reasons: no approval from an author; no approval from a third party; concerns about the data.

## Abbreviations

2-ME: Beta-mercaptoethanol
A1AT: Alpha-1 antitrypsin
aCGH: Array comparative genome hybridization
Cas: Clustered associated
CF: Cystic fibrosis
CFTR: Cystic fibrosis transmembrane conductance regulator
CGH: Comparative genome hybridization
CRISPr: Clustered regularly interspaced palindromic repeats
DSB: Double strand break
dsDNA: Double-stranded DNA
EB: Embryoid body
FGF2: Fibroblast growth factor 2
FIAU: 1-(2-deoxy-2-fluoro-1-D-arabinofuranosyl)-5-iodouracil
HDR: Homology-directed repair
hES: Human embryonic stem
hIPS: Human induced pluripotent stem
HR: Homologous recombination
HR: Homologous recombination
iPS: Induced pluripotent stem cells
NHEJ: Non-homologous end-joining
ORF: Open reading frame
PCR: Polymerase chain reaction
ROCK: Rho-associated, coiled-coil-containing protein kinase
RVD: Repeat variable domain
TALEN: Transcription activator-like effector nuclease
Tk: Tyrosin kinase
ZFN: Zinc-finger nuclease
